The article "Long noncoding RNA MLK7-AS1 promotes ovarian cancer cells progression by modulating miR-375/YAP1 axis" was retracted in 2020. Reasons: errors in the images; unreliable results or conclusions.

# Long noncoding RNA MLK7-AS1 promotes ovarian cancer cells progression by modulating miR-375/YAP1 axis

**DOI:** 10.1186/s13046-018-0910-4

**Published:** 2018-09-24

**Authors:** Huan Yan, Hong Li, Pengyun Li, Xia Li, Jianjian Lin, Linlin Zhu, Maria A. Silva, Xiaofang Wang, Ping Wang, Zhan Zhang

**Affiliations:** 1 Department of Obstetrics and Gynecology, The Third Affiliated Hospital of Zhengzhou University, Zhengzhou, Henan People’s Republic of China; 2 Department of Pathology and Laboratory Medicine, University of Tennessee Health Science Center, Memphis, TN USA; 3 Department of Clinical Laboratory, The Third Affiliated Hospital of Zhengzhou University, No. 7 Front Kangfu Street, Zhengzhou, 450052 Henan People’s Republic of China; 4 Department of Bioscience, University of Tennessee Health Science Center, Memphis, TN USA; 5 Collaborative Innovation Center of Molecular Diagnosis and Laboratory Medicine, Xinxiang Medical University, Xinxiang, Henan People’s Republic of China; 6 Department of Reproductive Medicine Center, the People’s Hospital of Henan Province, Zhengzhou, Henan People’s Republic of China

**Keywords:** LncRNA, MLK7-AS1, Ovarian cancer, miR-375, YAP1, Slug

## Abstract

**Background:**

Long noncoding RNAs (LncRNAs) have been reported to be abnormally expressed in human ovarian cancer and associated with the proliferation and metastasis of cancer cells. The objective of this study was to investigate the role and the underlying mechanisms of LncRNA MAP3K20 antisense RNA 1 (MLK7-AS1) in ovarian cancer.

**Methods:**

The expression level of MLK7-AS1 was investigated in human ovarian cancer tissues and cell lines. The effects of MLK7-AS1 knockdown on ovarian cancer cell proliferation, migration, invasion and apoptosis were evaluated in vitro using MTT, colony formation assays, wound healing assays, transwell assays and flow cytometry. Furthermore, the in vivo effects were determined using the immunodeficient NSG female mice. Luciferase reporter assays were employed to identify interactions among MLK7-AS1 and its target genes.

**Results:**

In the current study, MLK7-AS1 was specifically upregulated in ovarian cancer tissues and cell lines. Knockdown of MLK7-AS1 inhibited the ability of cell migration, invasion, proliferation, colony formation and wound healing, whereas promoted cell apoptosis in vitro. By using online tools and mechanistic analysis, we demonstrated that MLK7-AS1 could directly bind to miR-375 and downregulate its expression. Besides, MLK7-AS1 reversed the inhibitory effect of miR-375 on the growth of ovarian cancer cells, which might be involved in the upregulation of Yes-associated protein 1 (YAP1) expression. Moreover, knockdown MLK7-AS1 expression inhibited primary tumor growth in ovary and metastatic tumors in multiple peritoneal organs including liver and spleen in vivo, which were partly abolished by miR-375 inhibition. Mechanically, we found that MLK7-AS1 modulated the epithelial-mesenchymal transition (EMT) process by interacting with miR-375/YAP1 both in vivo and vitro, which promoted the expression of Slug.

The article "Long noncoding RNA MLK7-AS1 promotes ovarian cancer cells progression by modulating miR-375/YAP1 axis" was retracted in 2020. Reasons: errors in the images; unreliable results or conclusions.

**Conclusions:**

Taken together, our study showed for the first time that MLK7-AS1 interacted with miR-375 to promote proliferation, metastasis, and EMT process in ovarian cancer cells through upregulating YAP1.

## Background

Long non-coding (Lnc) RNAs are subjectively defined to be longer than 200 nucleotides and lack a conserved open reading frame and deeply involved in cellular activities such as cell growth, proliferation, apoptosis, epithelial-mesenchymal transition (EMT), metabolism, and drug resistance [1–3]. Recently, accumulating shreds of evidence suggested that dysfunction of LncRNAs were associated with human cancer, especially the circulating LncRNAs, which were stable and accessible and were considered potential candidate prognostic markers in some types of cancer. For example, Wang et al. demonstrated that serum LncRNA HOTAIR might serve as a potential biomarker for the diagnosis of esophageal squamous cell carcinoma. Zeng et al. found that upregulation of LncRNA DQ786243 was associated with poor prognosis and promoted tumor progression in hepatocellular carcinoma. Zhang et al. reported LncRNA TP73-AS1 interacted with miR-142 to modulate brain glioma growth through HMGB1/RAGE Pathway [4–6]. However, the exact contributions of LncRNAs to ovarian cancer remain largely unknown.

Mixed lineage kinase 7 (MLK7) is a mitogen-activated protein kinase kinase kinase (MAP3K) member, and the overexpression of MLK7 in cardiac myocytes activated SAPK/JNK1, ERK and p38 signaling pathways [7–9]. LncRNA MAP3K20 antisense RNA 1 (MLK7-AS1) has been recently identified as a novel oncogene in cancer. To date, in our knowledge, only one study has evaluated the role of MLK7-AS1 in cancer cells’ proliferation. Quan et al. found that MLK7-AS1 was upregulated in gastric cancer tissues, and the higher MLK7-AS1 level was an independent factor for poor prognosis of gastric cancer [10]. Besides, they reported that knockdown of MLK7-AS1 significantly inhibited cell proliferation and induced apoptosis in gastric cancer cells. However, the MLK7-AS1 expression level in ovarian cancer has not yet been reported, and its precise role in ovarian cancer remains to be elucidated.

Yes-associated protein 1 (YAP1), a 65-kDa proline-rich phosphoprotein, is one of the transcription co-activator which is regulated by the Hippo pathway [11–13]. Recently, YAP1 has been suggested to be a potent oncogene, and it was found to be elevated in several types of cancers. Zhu et al. demonstrated LncRNA UCA1 desensitized breast cancer cells to trastuzumab by impeding miR-18a repression of YAP1 [14]. Xu et al. showed that miR-622 suppressed the proliferation of glioma cells by targeting YAP1 [15]. Mou et al. found LncRNA ATB functioned as a competing endogenous RNA to promote YAP1 by sponging miR-590-5p in malignant melanoma [16]. In addition, YAP1 is also implicated in the EMT program in diverse cancers including liver, colon, prostate, ovarian, and breast cancers [17–19]. However, YAP1 expression level and the correlation with MLK7-AS1 in ovarian cancer have rarely been reported.

The article "Long noncoding RNA MLK7-AS1 promotes ovarian cancer cells progression by modulating miR-375/YAP1 axis" was retracted in 2020. Reasons: errors in the images; unreliable results or conclusions.

There is an increasing focus on the interaction between LncRNAs and miRNAs in diverse cancers. For example, LncRNA TP73-AS1 promoted breast cancer cell proliferation through miR-200a-mediated TFAM inhibition [20]. Besides, an inverse relationship was found between lncRNA XIST and miR-101, and knockdown of lncRNA XIST exerted its effects through regulating miR-101 to modulate EZH2 expression [21]. Moreover, LncRNA DQ786243 interacted with miR-506 and promoted progression of ovarian cancer cells [22].

In this study, our results showed for the first time that MLK7-AS1 interacted with miR-375 to promote proliferation, metastasis, and EMT process in ovarian cancer cells through upregulating YAP1.

## Methods

### Tissue samples collection

Forty-five paired ovarian cancer specimens, corresponding adjacent non-tumor tissues, and serum samples were collected from patients who underwent tumor surgical resections in the Third Affiliated Hospital of Zhengzhou University from March 2015 to March 2018. The study was approved by the Clinical Research Ethics Committee of the Zhengzhou University (No. 2015–158), and the informed consent and written approvals were obtained from all of the patients. The clinicopathological characteristics were summarized in Table 1.

**Table 1:** Clinicopathological factors and MLK7-AS1 expression in ovarian cancer patients

Characteristics		Total number	MLK7-AS1 expression				*P*-value
			High		Low		
			*n*	%	*n*	%	
Age	< 50	24	12	50	12	50	0.224
	≥50	21	10	47.6	11	52.4	
CA199	< 40	22	13	59.1	9	40.9	0.312
	≥40	23	10	43.5	13	56.5	
Differentiation	Well	16	6	37.5	10	62.5	0.058
	Moderate	17	9	52.9	8	47.1	
	Poor	12	5	41.7	7	58.3	
Menopause	Pre-	20	8	40	12	60	0.145*
	Post-	25	13	52	12	48	
Depth of invasion	T1-T3	18	3	16.7	15	83.3	0.005*
	T4	27	17	63	10	37	
Lymph node metastasis	Absent (N0)	16	5	31.2	11	68.8	< 0.001*
	Present (N1-N3)	29	19	65.5	10	34.5	
Distant metastasis	Absent (M0)	15	2	13.3	13	86.7	0.023*
	Present (M1)	30	24	80	6	20	
TNM stage	I-II	16	4	25	12	75	< 0.001*
	III-IV	29	24	82.8	5	17.2	

The article "Long noncoding RNA MLK7-AS1 promotes ovarian cancer cells progression by modulating miR-375/YAP1 axis" was retracted in 2020. Reasons: errors in the images; unreliable results or conclusions.

### Cell culture

The human ovarian cancer cell lines SKOV3, OVCAR3, PEO1, A2780, 3AO, CAOV3 and normal human ovarian surface epithelial cells (HOSEPiCs) were purchased from the American Type Culture Collection (ATCC, Manassas, VA, USA). Cells were cultured in DMEM (HyClone; Logan, USA), containing 10% fetal bovine serum, 100 U/ml penicillin and 100 mg/ml streptomycin (Gibco; Thermo Fisher Scientific, Inc., Grand Island, NY).

### Cell transfection

The miR-375 mimics/inhibitor and cDNA (pcDNA)-3.1/YAP1 plasmids were synthesized by GenePharma (Shanghai, China). Knockdown of LncRNA MLK7-AS1 and YAP1 were achieved by using lentivirus containing LncRNA MLK7-AS1/YAP1 siRNA sequences (GeneCopoecia, Guangzhou, China). The transfections were conducted using the lipofectamine 2000 (Invitrogen, Carlsbad, CA) transfection reagent, followed by the protocol recommended by the manufacturer. We verified all constructions for sequence correctness via direct sequencing. After 48-h transfection, the cells were collected and used for further experiments.

### 3-(4,5-Dimethylthiazol-2-yl)-2, 5-diphenyltetrazolium bromide assay

Cells were seeded into 96-well plates at a density of 3 × 10^3^ cells per well with DMEM medium supplemented with 10% FBS for 24 h, and 15 μL (5 mg/mL) 3-(4,5-dimethylthiazol-2-yl)-2,5-diphenyltetrazolium bromide (MTT) was added into each well and incubated in the dark for 4 h. Then 150 μL of dimethylsulfoxide was added to each well and was measured at the optical density (OD) at 570 nm.

### Cell colony formation assay

Cells (600 cells/well) were seeded into 6-well plates with DMEM medium supplemented with 10% FBS and cultured for 14 days. Then, colonies were fixed with methanol at room temperature for 15 min and stained with 0.1% crystal violet for 15 min (Invitrogen, Carlsbad, CA), and the total number of visible colonies were counted.

### Cell apoptosis analysis

SKOV3, OVCAR3 and PEO1 cells transfected with si-NC or si-MLK7-AS1 were harvested and then were double stained with FITC-Annexin V and PI. The results were analyzed using Cell Quest 3.5 software (BD Biosciences, San Jose, CA). Cells were divided into viable cells, dead cells, early and late apoptotic cells.

### Cell migration and invasion assays

Cell migration and invasion assays were measured using transwell inserts (8 μM pore size, Costar, Cambridge, MA, USA). Cells were seeded in uncoated (for migration assays) or coated (for invasion assays) with 100 μL Matrigel (BD Biosciences) transwell inserts (with 250 μL FBS-free DMEM), while 750 μL DMEM medium containing 20% FBS was added to the bottom chamber of 24-well plates, and 24 h later, all the transwell inserts were fixed in 4% paraformaldehyde for 20 min and then stained with crystal violet staining (for migration assays) and hematoxylin and eosin (H&E) staining (for invasion assays). The cell numbers were counted in 3 random fields of each chamber under the microscope. All experiments were repeated three times.

The article "Long noncoding RNA MLK7-AS1 promotes ovarian cancer cells progression by modulating miR-375/YAP1 axis" was retracted in 2020. Reasons: errors in the images; unreliable results or conclusions.

### Wound healing assay

SKOV3, OVCAR3 and PEO1 cells transfected with si-NC or si-MLK7-AS1 were cultured in DMEM medium containing 10% FBS and maintained at 37 °C with 5% CO_2_ for 36–48 h until 90–100% confluent. Linear scratches were created on the cell layer using a 20 uL pipette tip, and cells were maintained in serum-free DMEM medium for 24 h. The wound healing process was observed under an optical microscope and analyzed using Image J software (Bethesda, USA).

### RNA extraction and qRT-PCR

Total RNA was extracted from human ovarian cancer tissues and ovarian cancer cells and reversely transcribed into cDNAs by using a Reverse Transcription Kit (Toyobo, Tokyo, Japan). SYBR Green Real time PCR Master Mix (Toyobo, Tokyo, Japan) was used and reagents were subjected to 95 °C for 60 s and then subjected to 40 cycles of 95 °C for 15 s, 60 °C for 15 s and 72 °C for 45 s. The primers of miR-142, miR-375, miR-218, miR-193a, miR-499 were purchased from Sangon (Inc, Shanghai, China). The primers for MLK7-AS1 were: 5′-TTACCAGACACAACCAACCCC-3′ (forward), 5′-ATCAGTCAGGCCCATTGGTTT-3′ (reverse). The primers for YAP1 were: 5’-TGACCCTCGTTTTGCCATGA-3′ (forward), and 5’-GTTGCTGCTGGTTGGAGTTG-3′ (reverse); The primers for Slug were: 5′- CGAACCCACACATTGCCTTG-3′ (forward), and 5’-GTGAGGGCAAGAGAA AGGCT-3′ (reverse); The primers for GAPDH were: 5′-AGCCACATCGCTCAGACAC-3′ (forward) and 5′-GCCCAATACGACCAAATCC-3′ (reverse). All the results were normalized to the GAPDH mRNA level. 2^-ΔΔCT^ method was performed to analysis all the target genes of the relative fold changes.

### Western blot assay

Equal amounts (70 μg) of protein lysate were separated by 10% sodium dodecyl sulfate polyacrylamide gel electrophoresis and transferred to nitrocellulose membranes. The membranes were blocked with 5% (*w*/*v*) nonfat milk in Tris-buffered saline with 0.1% Tween (TBST) for 1 h and incubated with a rabbit monoclonal primary antibody against E-cadherin (ab40772; 1:1000; Abcam), N-cadherin (ab195186; 1:8000; Abcam), vimentin (ab45939; 1:1000; Abcam), Slug (ab63568; 1:800; Abcam), YAP1 (ab205270; 1:600; Abcam) and rabbit polyclonal anti-GAPDH (ab9485; 1:4000; Abcam) overnight at 4 °C. After a incubation with the corresponding horseradish peroxidase (HRP)-conjugated anti-rabbit secondary antibody (Sigma, USA) at 37 °C for 1 h, the protein bands were visualized by the enhanced chemiluminescence (ECL) Plus kit (Beyotime, Shanghai, China). The blots were detected on Kodak film developer (Fujifilm, Japan).

The article "Long noncoding RNA MLK7-AS1 promotes ovarian cancer cells progression by modulating miR-375/YAP1 axis" was retracted in 2020. Reasons: errors in the images; unreliable results or conclusions.

### Luciferase-reporter assay

With the lipofectamine 2000 transfection reagent, SKOV3 cells cultured in 24-well plates were co-transfected with luciferase-reporter plasmids and miRNA-mimics/−inhibitor, as well as the purified respiratory syncytial virus (pRSV)-β-galactosidase vector (internal control). Cells were harvested 48 h after transfection and the luciferase activity was monitored using a GloMax 20/20 luminometer (Promega). The β-Galactosidase activity from the pRSV-β-galactosidase vector was used for normalization of the luminescence levels. O-nitrophenyl-β-galactoside (ONPG) colorimetric assays were performed to measure β-galactosidase activity. The β-Galactosidase activity was evaluated by the measurement of O-nitrophenol using an ELISA plate reader (Bio-Rad, Hercules, CA, USA) at a wavelength of 450 nm.

### In vivo xenograft experiments

Animal experiments were approved by the Institutional Committee for Animal Research. SKOV3 cells transfected with si-MLK7-AS1–1/si-MLK7-AS1–1+ miR-375-inhibitor, si-MLK7-AS1–2/ si-MLK7-AS1–2 + miR-375-inhibitor, or si-NC (1.4 × 10^6^ cells in 10 μL) were injected into the left side ovary of each 6-week-old immunodeficient NSG female mice. Tumor growth was examined every 7-day for 6 weeks. Tumor volumes were detected with the formula: tumor volume (mm^3^) = (length × width^2^)/2. Then all mice were sacrificed and tumors were resected for further experiments.

### Immunofluorescence staining assay

Ovarian cancer cells were incubated with blocking buffer (5% normal goat serum, 3% bovine serum albumin, and 0.1% Triton-X 100 in PBS) for 1 h. Primary antibodies to YAP1 (ab205270; 1:200; Abcam), E-cadherin (ab76055; 1:150; Abcam), vimentin (ab45939; 1:100; Abcam), Slug (ab27568; 1:150; Abcam), and PCNA (ab29; 1:100; Abcam) were incubated with the cells overnight. After three rinsing for 5 min with PBST, Alexa Fluor 568 (red, goat anti-rabbit), 488 (green, goat anti-rabbit) and 488 (green, goat anti-mouse) antibodies were applied (1200 dilution, Invitrogen, Thermo Fisher, USA) for 1 h at room temperature. Cell nuclei were counterstained with DAPI (Burlingame, CA). Images were taken using a Nikon Ti inverted fluorescence microscope.

### RNA immunoprecipitation (RIP) assay

RNA immunoprecipitation (RIP) experiments were performed using the Magna RIP RNA-Binding Protein Immunoprecipitation Kit (Millipore, Stafford, VA) according to the manufacturer’s instructions. The cells were scraped off and lysed in complete RIP lysis buffer for 30 min. Then, 100 μl of whole cell extract was incubated with RIP buffer containing magnetic beads conjugated with the anti-Ago2 antibody (Cell Signaling, Danvers, MA, USA) overnight at 4 °C. Normal mouse IgG (Millipore) was used as negative control. Finally, purified RNAs in the precipitates were used to determine YAP1 (ab205270; Abcam) and Slug (ab27568; Abcam) expression.

The article "Long noncoding RNA MLK7-AS1 promotes ovarian cancer cells progression by modulating miR-375/YAP1 axis" was retracted in 2020. Reasons: errors in the images; unreliable results or conclusions.

### Statistical analysis

Experimental results were presented as mean ± SD. Statistical differences were analyzed by SPSS 20.0 software with Student’s t-test or one-way ANOVA. Correlations were performed by Pearson’s correlation. *P* < 0.05 was considered significant.

## Results

### MLK7-AS1 was upregulated and predicted poor clinical prognosis in ovarian cancer

The expression levels of MLK7-AS1 in 45 patients with ovarian cancer specimens and paired adjacent non-tumor tissues were determined using qRT-PCR. As shown in Fig. 1a, MLK7-AS1 expression was significantly upregulated in ovarian cancer samples compared to adjacent non-tumor tissues (*P* < 0.001). Furthermore, MLK7-AS1 expression was significantly upregulated in serum of ovarian cancer patients (*n* = 45) compared with healthy controls (*n* = 45, *P* = 0.0047) (Fig. 1b). Importantly, serum levels of MLK7-AS1 were positively associated with those of MLK7-AS1 in ovarian cancer tumor tissue (r^2^ = 0.5358, *P* = 0.001; Fig. 1c). Finally, MLK7-AS1 was also overexpressed in ovarian cancer cell lines: SKOV3, OVCAR3, PEO1, and A2780 compared to the normal HOSEPiCs (Fig. 1d).

**Fig. 1:** Expression levels of MLK7-AS1 in ovarian cancer tissues, serum, and cell lines. (**a**) Expression levels of MLK7-AS1 were upregulated in ovarian cancer tissues compared with the adjacent non-tumor tissues (*n* = 45). (**b**) MLK7-AS1 expressions were upregulated in ovarian cancer serum samples (n = 45) compared with the healthy controls (n = 45*).* (**c**) Correlation of MLK7-AS1 expression levels in ovarian cancer tissue and serum (n = 45). (**d**) Expression levels of MLK7-AS1 in ovarian cancer cell lines. (**e**) Patients with high MLK7-AS1 expression had poorer overall survival (OS) rates than those with low MLK7-AS1 expression (n = 45). (F) MLK7-AS1 expression was an independent prognostic indicator for OS in ovarian cancer patients. (**g**) ROC curve analysis was applied to determine the diagnostic value of MLK7-AS1. (**h**) Serum MLK7-AS1 expression levels were downregulated in postoperative samples (*n* = 45). Data presented as the mean ± standard deviation (SD) of three independent experiments. *P < 0.05, **P < 0.01

### Correlation of MLK7-AS1 expression with clinicopathological characteristics

Next, we analyzed the relationship between MLK7-AS1 expression and the clinical features of ovarian cancer. According to MLK7-AS1 expression levels obtained by qRT-PCR, we divided the 45 ovarian cancer patients into a relatively high MLK7-AS1 expression group (*n* = 27, 1.5-fold higher than normal tissues) and relatively low MLK7-AS1 expression group (*n* = 18). Patients with relatively high MLK7-AS1 expression exhibited a significant association deeper invasion (*P* = 0.005), worse lymphatic metastasis (*P* < 0.001), distant metastasis (*P* = 0.023), and advanced TNM stage (*P* < 0.001). However, there was no significant association between MLK7-AS1 expression and age, menopause, CA199 levels, or differentiation (Table 1).

The article "Long noncoding RNA MLK7-AS1 promotes ovarian cancer cells progression by modulating miR-375/YAP1 axis" was retracted in 2020. Reasons: errors in the images; unreliable results or conclusions.

### Upregulation of MLK7-AS1 was associated with poor prognosis in patients with ovarian cancer

Kaplan-Meier analysis and the log-rank test were used to analyze the relationship between MLK7-AS1 expression and patient survival. We found that the 5-year overall survival (OS) was significantly lower in patients with high MLK7-AS1 expression than in those with low MLK7-AS1 expression (*P* = 0.007; Fig. 1e).

Univariate analysis revealed that TNM stage (*P* < 0.001), depth of invasion (*P* = 0.021), lymph node metastasis (*P* = 0.030), distant metastasis (*P* = 0.014) and MLK7-AS1 expression levels (*P* = 0.001) were significantly correlated with OS (Table 2). In addition, multivariate analyses indicated that MLK7-AS1 expression (*P* = 0.017), TNM stage (*P* < 0.001), depth of invasion (*P* = 0.004), and lymph node metastasis (*P* = 0.023) were independent prognostic indicators for OS in ovarian cancer patients (Fig. 1f).

**Table 2:** Univariate and multivariable Cox proportional hazard regression analyses for overall survival

Variable	Univariate analysis				Multivariate analysis			
	HR	95% CI		*P*-value	HR	95% CI		*P*-value
Depth of invasion	2.012	1.802	2.312	0.021*	2.089	1.818	2.359	0.004*
Lymph node metastasis	1.910	1.610	2.016	0.030*	2.000	1.760	2.240	0.023*
Distant metastasis	1.524	1.366	1.681	0.014*				
TNM stage	1.934	1.689	2.234	< 0.001*	2.200	1.846	2.554	< 0.001*
MLK7-AS1	2.689	2.329	3.081	0.001*	2.975	2.554	3.396	0.017*

*HR* relative risk, 95% CI:95% confidence interval. *Statistically significant *P* < 0.05

### ROC curve of serum MLK7-AS1 level in the diagnosis of ovarian cancer

We further analyzed the ROC curve of serum MLK7-AS1 levels to assess its diagnostic value and found that serum MLK7-AS1 level could differentiate ovarian cancer patients from healthy controls (Fig. 1g), with an area under the curve (AUC) of 0.9565 (95% confidence interval [CI]: 0.915–0.998, *P* < 0.001). MLK7-AS1 may be an effective predictor for ovarian cancer diagnosis, with an optimal cut-off value of 2.39 (sensitivity, 86.7%; specificity, 71.1%). Moreover, postoperative serum samples from 45 patients were collected 1 month after surgery. The expression levels of serum MLK7-AS1 in postoperative specimens significantly decreased compared with those in preoperative samples (*P* < 0.001; Fig. 1h).

The article "Long noncoding RNA MLK7-AS1 promotes ovarian cancer cells progression by modulating miR-375/YAP1 axis" was retracted in 2020. Reasons: errors in the images; unreliable results or conclusions.

### Determination of the optimal interference sequence of si-MLK7-AS1

As shown in Fig. 2a, si-MLK7-AS1–1, si-MLK7-AS1–2, and si-MLK7-AS1–3 and negative control siRNA (si-NC) were transfected into SKOV3, OVCAR3 and PEO1 cells and the transfection efficiency was verified using qRT-PCR. The interference efficiency of si-MLK7-AS1–1 and si-MLK7-AS1–2 were higher rendering them as the optimal interference sequences (*P* < 0.01).

**Fig. 2:** The role of MLK7-AS1 in regulating ovarian cancer cell proliferation, colony formation, and apoptosis. (**a**) Comparison of interference efficiency of three MLK7-AS1 small interfering RNA sequences. (**b**) Cell growth viability was assayed in SKOV3, OVCAR3, and PEO1 cells transfected with si-NC, si-MLK7-AS1–1 or − 2 using MTT at 0 h, 24 h, 48 h, 72 h and 96 h time point. (**c**) Knockdown of MLK7-AS1 suppressed colony formation in SKOV3, OVCAR3, and PEO1 cells. (**d**) Cell apoptosis analysis was performed using flow cytometry. (**e**) Apoptosis related markers: Bcl-2, Bax, Bak and cleaved caspase 3 were detected using western blot assay in SKOV3, OVCAR3, and PEO1 cells transfected with si-NC, si-MLK7-AS1–1 or − 2. Data presented as mean ± SD of three independent experiments. *P < 0.05, **P < 0.01

### MLK7-AS1 knockdown suppressed proliferation in ovarian cancer cells

To investigate the role of MLK7-AS1 in ovarian cancer cells, MTT assay was performed, and the results showed that cell proliferation was significantly inhibited in the si-MLK7-AS1–1 and si-MLK7-AS1–2 transfected groups compared with that in the si-NC transfected group (Fig. 2b; *P* < 0.01). Similarly, colony formation assay revealed that cell colonies generated in the si-MLK7-AS1–1 and si-MLK7-AS1–2 transfected groups obviously decreased than that in the si-NC transfected group (Fig. 2c; *P* < 0.05).

Then, to further determine whether knockdown of MLK7-AS1 inhibited cell proliferation of ovarian cancer through changing cell apoptosis, flow cytometric analysis was used in our study, and cell apoptosis analysis indicated that the cell apoptosis rates in the si-MLK7-AS1–1 and si-MLK7-AS1–2 transfected groups were higher compared to that in the si-NC transfected group (Fig. 2d; *P* < 0.05). In addition, apoptosis related markers Bcl-2, Bax, Bak and cleaved caspase 3 were detected using western blot assay after knockdown of MLK7-AS1. We found that MLK7-AS1 knockdown decreased the Bcl-2 expression and increased the Bax, Bak and cleaved caspase 3 expression levels (Fig. 2e). Therefore, knockdown of MLK7-AS1 inhibited cell proliferation and induced cell apoptosis in ovarian cancer cells.

The article "Long noncoding RNA MLK7-AS1 promotes ovarian cancer cells progression by modulating miR-375/YAP1 axis" was retracted in 2020. Reasons: errors in the images; unreliable results or conclusions.

### MLK7-AS1 knockdown inhibited migration and invasion in ovarian cancer cells

Transwell assays were then performed to monitor the migration and invasion function of ovarian cancer cells in response to MLK7-AS1 knockdown. Results showed that MLK7-AS1 knockdown specifically suppressed the migration and invasion ability of SKOV3, OVCAR3 and PEO1 cells in vitro (Fig. 3a, b and c; *P* < 0.01). Similar results were obtained following a wound healing assay. Wound healing in SKOV3, OVCAR3 and PEO1 cells was significantly impaired in response to MLK7-AS1 knockdown compared to the si-NC transfected group (Fig. 3d, e and f; *P* < 0.01).

**Fig. 3:** The role of MLK7-AS1 in regulating ovarian cancer cell migration, invasion and wound healing. (**a**, **b**, **c**) Transwell assays were used to measure the effect of MLK7-AS1 knockdown on cell migration and invasion in SKOV3, OVCAR3, and PEO1 cells. (**d**, **e**, **f**) Wound healing assay was performed in SKOV3, OVCAR3, and PEO1 cells following transfection with si-NC and si-MLK7-AS1. The data were presented as mean ± SD of three independent experiments. The statistical results were shown on the right panel. **P < 0.01

### Candidate miRNAs scanning and verification

By using online tools including miRcode and Targetscan, we scanned out several candidate miRNAs that could bind with MLK7-AS1 and 3’UTR of YAP1. Combined with previous studies, we chose 5 candidate miRNAs which were reported to be related to tumorigenesis: miR-142, miR-375, miR-218, miR-193a, miR-499. To verify the interaction of MLK7-AS1 with candidate miRNAs, si-RNA or si-MLK7-AS1 was transfected into SKOV3, OVCAR3 and PEO1 cells, and then the mRNA levels were detected using qRT-PCR. Results showed that among the expressions of 5 candidate miRNAs, the level of miR-375 were the most strongly upregulated by MLK7-AS1 knockdown (Fig. 4a, b and c; *P* < 0.01).

**Fig. 4:** Candidate miRNAs scanning, verification and its correlation with MLK7-AS1. (**a**, **b**, **c**) si-NC, si-MLK7-AS1–1, or − 2 was transfected into SKOV3, OVCAR3, and PEO1 cells, and then the expression levels of 5 candidate miRNAs were monitored using qRT-PCR. (**d**) MLK7-AS1 interacted with miR-375 by directly targeting. (**e**) miR-375 expression was significantly upregulated after MLK7-AS1 knockdown. (**f**) MLK7-AS1 mRNA expression was significantly downregulated in response to miR-375 overexpression while upregulated in response to miR-375 inhibition. (**g**, **h**, **i**) si-MLK7-AS1 or/and miR-375-inhibitor was transfected into SKOV3, OVCAR3 and PEO1 cells, and the transfection efficiency was verified using qRT-PCR. (**j**, **k**, **l**) MTT results showed that MLK7-AS1 were significantly downregulated in si-MLK7-AS1–1 or − 2 group compared to the si-NC group, while the effects were reversed in miR-375 inhibition cotransfected groups. The data were presented as mean ± SD of three independent experiments. *P < 0.05, **P < 0.01

To confirm the predicted binding site of miR-375 to MLK7-AS1, both a wild-type (wt)-MLK7-AS1 and a mutant (mut)-MLK7-AS1 3′-UTR luciferase-reporter vector were constructed and transfected into SKOV3 cells, by sequentially mutating the two predicted miR-375-binding sites in the MLK7-AS1 3′-UTR (Fig. 4d). Then, wt-MLK7-AS1 and mut-MLK7-AS1, as well as mimics-NC/miR-375 mimics or inhibitor-NC/miR-375 inhibitor luciferase reporter vectors were co-transfected into SKOV3 cells, respectively. Results showed that the luciferase activity of the wt-MLK7-AS1 3′-UTR was obviously downregulated by miR-375-mimic transfection, while was significantly upregulated by miR-375-inhibitor transfection (*P* < 0.01). However, no significant differences of the luciferase activity of mut-MLK7-AS1 reporter were shown in cells transfected with miR-375-mimics or miR-375-inhibitor, suggesting the sequence-specific binding of miR-375 to MLK7-AS1 (*P* < 0.01).

The article "Long noncoding RNA MLK7-AS1 promotes ovarian cancer cells progression by modulating miR-375/YAP1 axis" was retracted in 2020. Reasons: errors in the images; unreliable results or conclusions.

### The correlation between MLK7-AS1 and miR-375 in ovarian cancer cells

To investigate whether MLK7-AS1 could interact with miR-375 and regulate progression in ovarian cancer cells, we detected the association between MLK7-AS1 and miR-375. Initially, qRT-PCR showed that miR-375 expression was notably upregulated after MLK7-AS1 knockdown in comparison with the si-NC transfected group (Fig. 4e; *P* < 0.01). Then, miR-375 overexpression or inhibition was transfected into SKOV3, OVCAR3 and PEO1 cells, and the transfection efficiency was verified using qRT-PCR. We found MLK7-AS1 mRNA expression was significantly downregulated in response to miR-375 overexpression while upregulated in response to miR-375 inhibition. (Fig. 4f; *P* < 0.01). Then, si-NC/si-MLK7-AS1 and inhibitor-NC/miR-375 inhibitor were co-transfected into SKOV3, OVCAR3 and PEO1 cell lines. The results showed that the inhibitory effect of si-MLK7-AS1 on SKOV3, OVCAR3 and PEO1 cell growth was partly restored by miR-375 inhibition (Fig. 4g, h and i; *P* < 0.01). Similar results were observed in cell MTT assay: the growth of SKOV3, OVCAR3 and PEO1 cell lines was significantly decreased in response to MLK7-AS1 knockdown by si-MLK7-AS1, while it was increased in response to miR-375 inhibition; the inhibitory effect of si-MLK7-AS1 on cell growth was partly abolished by miR-375 inhibition (Fig. 4j, k and l; *P* < 0.01). Therefore, we presumed that MLK7-AS1 might promote tumorigenesis and growth by suppressing the activity of miR-375 in ovarian cancer.

The article "Long noncoding RNA MLK7-AS1 promotes ovarian cancer cells progression by modulating miR-375/YAP1 axis" was retracted in 2020. Reasons: errors in the images; unreliable results or conclusions.

### YAP1 promoted the progression of ovarian cancer cells

Emerging evidence has proved the role of YAP1 in cancer cell progression. Initially, our research showed that the mRNA and protein expression levels of YAP1 were obviously elevated in ovarian cancer tissues compared with adjacent normal tissues (Fig. 5a and b; *P* < 0.01). Besides, YAP1 mRNA and protein expressions were greatly reduced by MLK7-AS1 knockdown in ovarian cancer cell lines (Fig. 5c and d; *P* < 0.01); Moreover, we further immunostained SKOV3, OVCAR3, and PEO1 cells with antibodies to YAP1, and the immunofluorescence of YAP1 was downregulated in MLK7-AS1 knockdown groups compared to that in the si-NC transfected group (Fig. 5e and f; *P* < 0.01). Interestingly, MLK7-AS1 mRNA expression was notably decreased by YAP1 knockdown in ovarian cancer cell lines (Fig. 5g; *P* < 0.01).

**Fig. 5:** The expression levels and the correlation between MLK7-AS1 and YAP1. (**a**, **b**) The mRNA and protein expression levels of YAP1 were significantly elevated in ovarian cancer tissue samples compared with adjacent normal tissues. (**c**, **d**) The mRNA and protein expression levels of YAP1 were significantly decreased by the MLK7-AS1 knockdown in ovarian cancer cell lines. (**e**, **f**) YAP1 levels were greatly decreased by the MLK7-AS1 knockdown in ovarian cancer cell lines using immunofluorescence. (**g**) MLK7-AS1 mRNA expression greatly reduced by YAP1 knockdown in SKOV3, OVCAR3, and PEO1 cell lines. (**h**) pcDNA3.1/YAP1 was transfected into SKOV3, OVCAR3, and PEO1 cell lines to get YAP1 overexpression, and the effects were verified using western blot. (**i**) The inhibition effects of MLK7-AS1 knockdown on cell growth were partly reversed by YAP1 overexpression using MTT assay. The data were presented as mean ± SD of three independent experiments. *P < 0.05, **P < 0.01

### MLK7-AS1 regulated ovarian cancer cell growth through targeting YAP1

We further investigated whether MLK7-AS1 regulated ovarian cancer cell growth through targeting YAP1. The plasmids of cDNA (pcDNA)-3.1/YAP1 were transfected into SKOV3, OVCAR3, and PEO1 cell lines to achieve YAP1 overexpression, which was verified using western blot (Fig. 5h; *P* < 0.01).

Then, si-NC/si-MLK7-AS1 and pcDNA3.1/YAP1 were co-transfected into SKOV3, OVCAR3, and PEO1 cell lines. MTT assay was used to determine the cell growth. Results showed that the growth of three ovarian cancer cell lines were significantly decreased in response to MLK7-AS1 knockdown by si-MLK7-AS1, while it was increased in response to YAP1 overexpression; the inhibitory effects of si-MLK7-AS1 on SKOV3, OVCAR3, and PEO1 cell growth were partly restored by YAP1 overexpression (Fig. 5i; *P* < 0.01). In sum, MLK7-AS1 regulated ovarian cancer-cell growth through targeting YAP1.

The article "Long noncoding RNA MLK7-AS1 promotes ovarian cancer cells progression by modulating miR-375/YAP1 axis" was retracted in 2020. Reasons: errors in the images; unreliable results or conclusions.

### MLK7-AS1 interacted with miR-375 and promoted progression of ovarian cancer through targeting YAP1

We further investigated whether miR-375 could regulate YAP1 expression in ovarian cancer cells. Similarly, the wt-YAP1 or mut-YAP1′-UTR luciferase reporter vectors, as well as mimics-NC/miR-375-mimics or inhibitor-NC/miR-375-inhibitor were co-transfected into SKOV3 cells, respectively. The activity of the wt-YAP1 3’UTR vector was significantly downregulated in the miR-375-mimics group compared to the mimics-NC group, while upregulated in the miR-375-5p-inhibitor transfected group compared to the inhibitor-NC group (Fig. 6a and b; *P* < 0.01). However, no significant differences of the luciferase activity of mut-YAP1 reporter were found in cells transfected with miR-375-mimics or miR-375-inhibitor. Taken together, these data indicated that miR-375 negatively regulated YAP1 by targeting to its 3’UTR.

**Fig. 6:** MLK7-AS1 interacted with miR-375 and promoted progression of ovarian cancer cell through targeting YAP1. (**a**) YAP1 was predicted to be a target gene of miR-375 by TargetScan. (**b**) miR-375 regulated YAP1 expression by direct targeting using luciferase assay. (**c**) miR-375 levels were significantly decreased in human ovarian cancer tissues compared with adjacent non-tumor tissues. (**d**, **e**, **f**) The qRT-PCR assay showed that mRNA expressions of YAP1 were downregulated by miR-375 overexpression while upregulated by miR-375 inhibition in SKOV3, OVCAR3, and PEO1 cell lines. (**g**, **h**, **i**) Western blot assay showed that protein expressions of YAP1 were downregulated by miR-375 overexpression while upregulated by miR-375 inhibition in SKOV3, OVCAR3, and PEO1 cell lines. 1, mimics-NC; 2, miR-375-mimics; 3, inhibitor-NC; 4, miR-375-inhibitor. (**j**, **k**, **l**) The inhibitory function of MLK7-AS1 knockdown on YAP1 protein level was partially restored by the miR-375 inhibition. The data were presented as mean ± SD of three independent experiments. *P < 0.05, **P < 0.01

Our research found showed that the mRNA expression level of miR-375 was obviously decreased in ovarian cancer tissue samples compared with adjacent normal tissues (Fig. 6c; P < 0.01). Besides, qRT-PCR (Fig. 6d, e and f) and western blot assays (Fig. 6g, h and i) showed that mRNA and protein expressions of YAP1 were downregulated by miR-375 overexpression while upregulated by miR-375 inhibition in SKOV3, OVCAR3, and PEO1 cell lines.

The article "Long noncoding RNA MLK7-AS1 promotes ovarian cancer cells progression by modulating miR-375/YAP1 axis" was retracted in 2020. Reasons: errors in the images; unreliable results or conclusions.

Then, we further validated whether MLK7-AS1 could interact with miR-375 and promote progression of ovarian cancer through targeting YAP1. As determined by western blot assay, YAP1 protein expression levels were downregulated by si-MLK7-AS1 transfection, whereas the levels were significantly upregulated by miR-375-inhibitor transfection in SKOV3, OVCAR3, and PEO1 cell lines; which suggested that the inhibitory function of MLK7-AS1 knockdown on YAP1 mRNA and protein levels were partially restored by miR-375 inhibitor (Fig. 6j, k and l; *P* < 0.01).

### MLK7-AS1 interacted with miR-375 to promote the EMT process in ovarian cancer cells

EMT is a key process for cancer cell invasion and migration. Cells undergoing EMT assume a variety of mesenchymal-like properties: enhanced migratory capacity, invasiveness, heightened resistance to apoptosis. To detect whether expression levels of MLK7-AS1 regulated EMT process in ovarian cancer cells, we immunostained SKOV3, OVCAR3 and PEO1 cells with E-cadherin and vimentin, respectively. Interestingly, E-cadherin (Fig. 7a) was upregulated and vimentin (Fig. 7b) was downregulated in the MLK7-AS1–1 or MLK7-AS1–2 knockdown group compared to the si-NC group, while the effects were reversed by miR-375 inhibition. In sum, these results suggested that MLK7-AS1 interacted with miR-375 to promote the EMT process in vitro.

**Fig. 7:** YAP1 promoted the EMT process by inducing Slug transcription. (**a**, **b**) E-cadherin and vimentin expression levels were determined when MLK7-AS1 knockdown or/and miR-375 inhibition in SKOV3, OVCAR3, and PEO1 cell lines using immunofluorescence. (**c**) By using gene sequence analysis, a putative binding site of the YAP1 in the promoter of Slug was found. (**d**, **e**) Slug protein and mRNA levels were increased in SKOV3, OVCAR3, and PEO1 cells when YAP1 was overexpressed. (**f**, **g**) Slug protein and mRNA levels were decreased in SKOV3, OVCAR3, and PEO1 cells when YAP1 was knockdown. (**h**, **i**, **j**) Slug expression levels were distinctly higher in tumor tissues than in adjacent non-tumor tissues using H&E, immunofluorescence, and qRT-PCR, respectively. (**k**) Slug expressions were determined when YAP1 was overexpressed or knockdown using immunofluorescence. (**l**, **m**, **n**) A RIP assay was performed to examine whether YAP1 and Slug were in the same RNA-induced silencing complex. (**o**) YAP1 regulated Slug expression by direct targeting using a luciferase assay. The data were presented as mean ± SD of three independent experiments. *P < 0.05, **P < 0.01

The article "Long noncoding RNA MLK7-AS1 promotes ovarian cancer cells progression by modulating miR-375/YAP1 axis" was retracted in 2020. Reasons: errors in the images; unreliable results or conclusions.

### YAP1 promoted the EMT process by inducing slug transcription

We further detected the underlying mechanisms of the MLK7-AS1/miR-375 axis in regulating EMT in ovarian cancer cells. EMT inducers converge to activate transcription factors, including three families, Slug, Twist and ZEB, directly or indirectly suppress the E-cadherin promoter [23]. Slug is a member of the Snail family and can repress E-cadherin expression and trigger EMT, and Slug was reported to be involved in malignant transformation and metastatic progression in numerous cancers [24].

By using gene sequence analysis, we found a putative binding site of the YAP1 in the promoter of Slug (Fig. 7c). In addition, we found that overexpression of YAP1 upregulated protein and mRNA expression levels of Slug in SKOV3, OVCAR3 and PEO1 cells (Fig. 7d and e; *P* < 0.01). Inversely, knockdown expression of YAP1 reduced protein and mRNA expressions of Slug (Fig. 7f and g; *P* < 0.01). In particular, Slug expression levels were much higher in tumor tissues than in adjacent tissues using H.E. staining, immunofluorescence staining and qRT-PCR, respectively (Fig. 7h, i and j; *P* < 0.01); As we proved before, YAP1 was also highly expressed in tumor tissues. Thus, these results suggested that the ability of YAP1 to promote EMT might be associated with the activation of Slug expression.

Slug can suppress E-cadherin expression by directly binding to the E-cadherin promoter; thus, it is a mediator of the EMT program in many epithelial tumors, such as in lung cancer progression. Therefore, we tested the possibility that Slug is a mediator of EMT in YAP1 overexpressed ovarian cancer cells and that Slug is the target gene of YAP1. Firstly, the immunofluorescence staining results showed that overexpressing YAP1 promoted the expression of Slug in the nucleus, while silencing YAP1 also inhibited Slug expression levels in the nucleus in SKOV3, OVCAR3 and PEO1 cells compared with those in the control group (Fig. 7k; *P* < 0.01); Next, a RIP assay was performed to examine whether YAP1 and Slug are in the same RNA-induced silencing complex. It was revealed that YAP1 and Slug were enriched in Ago2 immunoprecipitates compared with the control IgG group in SKOV3, OVCAR3 and PEO1 cell lines (Fig. 7l, m, n; *P* < 0.01). Consistent with these results, luciferase assays showed that overexpressing YAP1 promoted the luciferase activity of the wt-Slug-Luc promoter, whereas overexpressing YAP1 had no influence on the luciferase activity of the mut-Slug-Luc promoter (Fig. 7o; *P* < 0.01); These results illustrated that Slug is a target gene of YAP1 and MLK7-AS1/miR-375/YAP1 axis might promote the EMT program by inducing Slug transcription and thus contribute to ovarian cancer.

The article "Long noncoding RNA MLK7-AS1 promotes ovarian cancer cells progression by modulating miR-375/YAP1 axis" was retracted in 2020. Reasons: errors in the images; unreliable results or conclusions.

### MLK7-AS1 interacted with miR-375 to promote tumor growth, metastasis and EMT process in vivo

To determine the effect of MLK7-AS1 on tumor growth in vivo, SKOV3 cells transduced with si-MLK7-AS1 were injected subcutaneously into immunodeficient NSG female mice. We found that tumors were obviously smaller in mice xenografted with MLK7-AS1 knockdown SKOV3 cells compared to control cells as shown by xenograft live animal imaging system. However, when miR-375-inhibitor and si-MLK7-AS1 cotransfected SKOVS cells were injected into mice, the MLK7-AS1 down-regulation effect on primary tumor growth was partly abolished (Fig. 8a and b). The mean volume and weight of the xenograft tumors were lower in the si-MLK7-AS1 group than in the si-NC group and this effect was also partly reversed by miR-375-inhibition treatment (Fig. 8c, d, e, and f). In addition, knockdown of MLK7-AS1 decreased the ability of primary tumors to metastasize to liver and spleen in vivo, moreover, the effects were abolished in miR-375-inhibition cotransfected group (Fig. 8g and h).

**Fig. 8:** MLK7-AS1 interacted with YAP1 to promote tumor growth, metastasis and EMT process in vivo. (**a**, **b**) Primary tumors in ovary were imaged at 6 weeks after injection by xenograft live animal imaging. (**c**, **d**) Tumor growth curves measured after injection of si-MLK7-AS1 or si-MLK7-AS1 + miR-375-inhibitor SKOV3 cells. Tumor size was evaluated using the average maximal luminescence from the mice. (**e**, **f**) Tumors from NSG mice xenografted with si-MLK7-AS1 or si-MLK7-AS1 + miR-375-inhibitor SKOV3 cells were dissected and weighed. (**g**) Knockdown of MLK7-AS1 suppressed the ability of primary tumors to metastasize to liver and spleen in vivo, moreover, the effects were abolished in the miR-375-inhibition cotransfected group. (**h**) H.E. stained sections of primary tumor in ovary, liver and spleen of NSG mice injected with si-MLK7-AS1 or si-MLK7-AS1 + miR-375-inhibitor SKOV3 cells. (**i**) Western blot analysis of E-cadherin, N-cadherin, vimentin, YAP1 and Slug in primary tumors of ovary. (**j**, **k, l**) The expressions of E-cadherin, vimentin, cell proliferation marker gene PCNA, YAP1 and Slug were determined using immunofluorescence in primary tumors of ovary. The data were presented as mean ± SD of three independent experiments. *P < 0.05, **P < 0.01

Then, to examine whether MLK7-AS1 expression regulated EMT process in tumor xenografts, EMT marker genes were detected using western blot assay in mice tumor tissues. As showed in Fig. 8i, n-cadherin, vimentin, Slug as well as YAP1 were downregulated, whereas E-cadherin was upregulated in tumors transfected with MLK7-AS1 knockdown SKOV3 cells compared to the controls, however, the MLK7-AS1 inhibition effect was partly abolished when miR-375-inhibition and MLK7-AS1-knockdown were cotransfected into SKOV3 cells.

The article "Long noncoding RNA MLK7-AS1 promotes ovarian cancer cells progression by modulating miR-375/YAP1 axis" was retracted in 2020. Reasons: errors in the images; unreliable results or conclusions.

Moreover, we further immunostained tumor sections with antibodies to E-cadherin, vimentin as well as cell proliferation marker gene PCNA. Interestingly, E-cadherin was upregulated, vimentin and PCNA were downregulated in the si-MLK7-AS1 group compared to the si-NC group; similarly, the MLK7-AS1 inhibition effect was partly abolished when miR-375-inhibitor and MLK7-AS1-knockdown were cotransfected into SKOV3 cells (Fig. 8j and k). Moreover, YAP1 and Slug protein and fluorescence expressions were decreased in the si-MLK7-AS1 group compared to the si-NC group, similarly, the inhibition effect was partly abolished when miR-375-inhibition was co-transfected, these results suggested that the ability of YAP1 to promote EMT might be associated with the activation of Slug expression in vivo (Fig. 8l).

Taken together, these results suggested that MLK7-AS1 interacted with miR-375 to promote tumor growth, metastasis and EMT process in vivo.

## Discussion

LncRNA MLK7-AS1 has been identified as one of the cancer-specific LncRNAs, its expression was significantly associated with the overall survival of patients with gastric cancer [5]. A recent study demonstrated that high MLK7-AS1 expression contributed to the proliferation and inhibited apoptosis of gastric cancer. Similarly, in the current study, we found that MLK7-AS1 expression levels were significantly elevated both in ovarian cancer tissues and in serums. Moreover, higher MLK7-AS1 expression was associated with poor survival and adverse clinical pathological characteristics including worse pathological T stage, more lymph node metastasis, distant metastasis and deeper invasion. Importantly, our results revealed that serum MLK7-AS1 levels could differentiate ovarian cancer patients from healthy controls. These results indicated that MLK7-AS1 can be regarded as a valuable diagnostic and prognostic marker for patients with ovarian cancer. Moreover, we found that knockdown of MLK7-AS1 obviously suppressed cell proliferation, colony formation, migration and invasion, while promoted cell apoptosis in ovarian cancer cell lines.

Ovarian cancer is one of the most lethal gynecological malignancies, with a five-year survival rate of only 30% due to intraperitoneal metastasis. Thus, to assess the function of MLK7-AS1 knockdown on tumor growth and metastasis in vivo, xenograft models were applied, and the results revealed that MLK7-AS1 knockdown specifically inhibited primary tumor growth in ovaries and metastatic tumors in multiple peritoneal organs including liver and spleen. This is the first time we proved the role of MLK7-AS1 expression in human ovarian cancer, which led us to propose that MLK7-AS1 may serve as a tumor promoter in ovarian cancer progression and metastasis.

miR-375 has been reported to express in various tumors, which shown to play a suppressive role in regulating tumor cells proliferation and apoptosis. Wang et al. found that miR-375 inhibited the invasion and migration of laryngeal squamous cell carcinoma synergistically via AKT-mediated EMT [25]. Yu et al. examined the suppression effect of miR-375 in the proliferation of HPV16-positive human cervical cancer cells [26]. Moreover, Quan et al. demonstrated that MLK7-AS1 exerted its oncogenic functions by epigenetically downregulating miR-375 [10]. In line with their studies, we observed a significant increase of miR-375 expression level by MLK7-AS1 knockdown in SKOV3, OVCAR3 and PEO1 cells. In the meantime, miR-375 inversely regulated MLK7-AS1 expression in ovarian cancer tissues, and a luciferase assay further confirmed the direct binding of miR-375-5p to MLK7-AS1. Moreover, miR-375 inhibition treatment partly abolished the suppression effects of MLK7-AS1 knockdown on primary ovary tumor growth as well as metastatic tumors in liver and spleen in vivo. Therefore, we assumed that MLK7-AS1 might suppress the activity of miR-375 through regulating its downstream target mRNAs in ovarian cancer.

The article "Long noncoding RNA MLK7-AS1 promotes ovarian cancer cells progression by modulating miR-375/YAP1 axis" was retracted in 2020. Reasons: errors in the images; unreliable results or conclusions.

As a major downstream target of the Hippo pathway, YAP1 has been reported to promote tumorigenesis via impacting on proliferation in a various tumor cell, such as colon, bladder and liver cancers [27–29]. In our study, we observed a higher expression of YAP1 in ovarian cancer tissues and cell lines. Besides, YAP1 protein expression in SKOV3, OVCAR3 and PEO1 cells were significantly decreased in response to MLK7-AS1 knockdown. Furthermore, when si-MLK7-AS1 and YAP1 overexpression plasmids were cotransfected into ovarian cancer cell lines, the inhibitory effects of si-MLK7-AS1 on cells growth were partly restored by YAP1 overexpression. These indicated that MLK7-AS1 might regulate YAP1 expression to modulate ovarian cancer cells’ proliferation.

Moreover, Hippo-YAP signaling pathway takes part in regulating apoptosis of cancer cells and has crosstalk with caspase3 and Bcl-2 signaling pathways. In this study, the apoptosis rate of ovarian cancer cells apparently increased when MLK7-AS1 was knockdown. Similarly, the expression levels of cleaved caspase3 and Bcl-2 family members (Bak, Bax) increased when MLK7-AS1 was interfered. This result reflected the association between caspase3 and Bcl-2 signaling pathways and hippo signaling pathway, and YAP could regulate the apoptosis rate of ovarian cancer cells through caspase3 and Bcl-2 signaling pathways.

The article "Long noncoding RNA MLK7-AS1 promotes ovarian cancer cells progression by modulating miR-375/YAP1 axis" was retracted in 2020. Reasons: errors in the images; unreliable results or conclusions.

As a potent oncogene, YAP1 has been confirmed as a target gene of several miRNAs. For example, miR-375 was found to be an important tumor suppressor in gastric cancer by targeting YAP1 [30]. Therefore, we further investigated whether miR-375 could directly regulate YAP1 in ovarian cancer. Interestingly, YAP1 protein expression was downregulated by miR-375 overexpression while upregulated by miR-375 inhibition in SKOV3, OVCAR3 and PEO1 cells. As expected, a luciferase assay further confirmed the direct binding of miR-375-5p to YAP1.

Since we confirmed the direct binding of miR-375-5p to YAP1 in ovarian cancer, and we have proved that MLK7-AS1 interacted with YAP1 to modulate ovarian cancer cells’ proliferation, migration and invasion. Therefore, we hypothesized that MLK7-AS1 might regulate YAP1 via miR-375. As proved by western blot assay, the inhibitory effects of MLK7-AS1 knockdown on YAP1 protein levels were partially restored by miR-375 inhibition. These data showed that MLK7-AS1 could regulate YAP1 through miR-375.

EMT is a process in which cancer cells lose their epithelial characteristics and acquire mesenchymal properties, thus promoting cell invasion and metastasis. The EMT process plays a crucial role during the progression of many types of cancers including human ovarian cancer [17, 23, 31]. Recent studies have demonstrated that LncRNAs are involved in regulation the EMT pathway [5, 32, 33]. In this study, our data also showed that knockdown of MLK7-AS1 upregulated epithelial maker expression levels but downregulated the expression levels of mesenchymal marker genes both in in vitro and *vivo*, while the suppression effects were partly reversed by miR-375-inhibition, indicating MLK7-AS1 might interact with miR-375 to promote cell proliferation via the EMT pathway in ovarian cancer cells.

Slug, a key EMT regulator, is best known for its role in orchestrating EMT programs associated with development [34, 35]. Recently, Yi Tang et al. suggested that Snai1 and Slug impacted stem cell functions and bone formation via cooperative interaction with YAP/TAZ [36], but whether there is a direct interaction between Slug and YAP1 that could induce EMT has not been described previously. In our study, we found that YAP1 induced the EMT process in ovarian cancer cells through promoting the transcription of Slug. These data suggest that the transcriptional regulation between YAP1 and Slug may impact ovarian cancer cell functions, which was consistent with previous research [37]; these actions deserve further investigation in the future.

The article "Long noncoding RNA MLK7-AS1 promotes ovarian cancer cells progression by modulating miR-375/YAP1 axis" was retracted in 2020. Reasons: errors in the images; unreliable results or conclusions.

## Conclusions

Taken together, we showed for the first time that MLK7-AS1 played pivotal roles in the aggressive biology of ovarian cancer, and our data indicated that LncRNA MLK7-AS1/miR-375/YAP1 axis contributed to tumor proliferation, metastasis and induced EMT in ovarian cancer cells. The present study might help with the exploration of new therapeutic strategies for the treatment of ovarian cancer.

## Abbreviations

LncRNA: Long non-coding RNA MLK7-AS1 Mixed lineage kinase 7 antisense RNA 1 YAP1 Yes-associated protein 1 miR-375 microRNA-375 siRNA Small interfering RNA 3′-UTR 3′-untranslated regions MTT 3-(4,5-dimethyl-2-thiazolyl)-2,5-dipheny EMT epithelial-to-mesenchymal transition OD optical density
